The article "Application of Three-Stage DEA Model Combined with BP Neural Network in Microfinancial Efficiency Evaluation" was published in 2022. Journal: Comput Intell Neurosci.

# Application of Three-Stage DEA Model Combined with BP Neural Network in Microfinancial Efficiency Evaluation

**DOI:** 10.1155/2022/8500662

**Published:** 2022-07-04

**Authors:** Jiale Yang, Xiang Li, Jie Mei, Liang Chen

**Affiliations:** ^1^International College, Guangxi University, Nanning 530004, China; ^2^School of Mathematics and Information Science, Guangxi University, Nanning 530004, China

## Abstract

The research performed here intends to explore the future development model of new rural financial institutions and determine the financial efficiency goals, thereby providing a huge stage for the development of new rural financial institutions. It applies data envelopment analysis (DEA) to assess financial efficiency to make up for the research gap. First, the relevant theories of rural finance are discussed. Then, some indicators are selected to build an evaluation system. In addition, the DEA method is used to evaluate the rural financial efficiency in Hebei Province by listing the input indexes and output indexes. After training, the backpropagation neural network (BPNN) model is designed and simulated to obtain the evaluation results. The research results show that before 2015, the comprehensive efficiency of Xingtai, Hengshui, Shijiazhuang, and Langfang showed a downward trend. After 2015, the comprehensive efficiency of all cities in Hebei Province tended to be stable, generally stable at about 0.95. It suggests that rural finance in Hebei Province has developed stably in recent years, and the overall efficiency of rural finance has been improved to a certain extent. The simulation results of BPNN demonstrate that the operation efficiency evaluation result of the poverty alleviation development model in the financial support industry is 0.6995, in the interval (0.6, 0.8). In addition, the model operation efficiency is better, indicating that the poverty alleviation development model of the financial support industry has achieved good results and promoted the development of poor rural areas. The research content can provide reference and inspiration for the continuous promotion of rural finance and the formulation and implementation of financial institution reform policies.

## 1. Introduction

A perfect and efficient rural financial market can significantly promote smooth consumption, reduce liquidity constraints, and then reduce poverty. Therefore, promoting the development of rural finance is an ideal poverty alleviation policy, thereby promoting the development of the rural economy. However, the results of theoretical research and empirical analysis in the past three decades show that the rural financial sector in developing countries is highly heterogeneous, the degree of financial repression and welfare losses for farmers and microenterprises is relatively serious, and the operation efficiency of rural financial markets is low. After a long period of financial system reform, the service situation of China's rural financial departments has been greatly improved, but there are still many problems to be solved. Rural finance is still a weak link that restricts the development of China's rural economy. The coverage rate of rural financial institutions is low, the internal management system is not perfect, and the service supply is insufficient. The No. 1 Central Document in 2019 made arrangements for the comprehensive deepening of rural reform, focusing on solving the problems of “rural stability, farmers' income increase, and agricultural growth.” It is imperative to deepen agrarian reform to win the battle against poverty. However, backward agricultural production and slow rural economic development still exist. Rural finance plays a critical role in rural economic growth [1, 2]. The service situation of China's rural financial sector has been dramatically improved after a period of system reform. Still, there are imperfect internal management systems, a lack of service supply, and low network coverage in rural financial institutions. The weak link restricts the development of China's rural economy [3]. To solve the above problems, China has attached great importance to reforming the rural financial system. In addition, the government is committed to increasing the adequate financial supply in the rural financial market to promote the sustainable and stable development of the rural economy.

The article "Application of Three-Stage DEA Model Combined with BP Neural Network in Microfinancial Efficiency Evaluation" was published in 2022. Journal: Comput Intell Neurosci.

With the development of new rural financial institutions, the financial efficiency of its subsystems is proposed. The key to developing new rural financial institutions lies in the efficiency of financial capital allocation. Only through effective financial resource allocation can the positive role of new rural financial institutions be brought into play to truly solve the problems encountered in rural economic development [4, 5]. Many scholars have carried out relevant research on financial efficiency to solve the problems in the operation of new rural financial institutions. Hein et al. [6] assessed whether the uniformity of financial metrics had an ordinal correlation with the sales ranking of the 500 largest companies corresponding to 2018 published by Exame magazine. To clarify this doubt, the author used the TOPSIS multicriteria method to evaluate the scale of financial indicators. The results showed that the companies' positioning in the sample changed. Luthfan et al. [7] noted that efficiency was an indicator of bank performance; a bank's efficiency was affected by how management manages risk. The author measured the impact of financing risk, operational risk, and liquidity risk on the level of efficiency. Efficiency was measured from operating income through the operating expenditure method. Through the statistical test, discussion and analysis, and financing risk, they found that operational risk and liquidity risk jointly affected the efficiency level.

The article "Application of Three-Stage DEA Model Combined with BP Neural Network in Microfinancial Efficiency Evaluation" was published in 2022. Journal: Comput Intell Neurosci.

Referring to the relevant literature, it can be found that the current research on rural financial efficiency mainly focuses on the efficiency of resource allocation, and there is a lack of targeted research for a particular region. In studying the pastoral financial efficiency process, it is essential to evaluate the level of financial efficiency and accurately grasp its influencing factors to determine the factors affecting rural finance. First, the related concepts and basic theories about rural finance are sorted out, which lays the foundation for the research content. Second, the current situation of rural economy and rural financial development in Hebei Province is analyzed. On the basis of the analysis, the data envelopment analysis (DEA) model is used to analyze and calculate the superefficiency value of rural financial efficiency in Hebei Province. Finally, taking the superefficiency value as the explained variable, by constructing a panel data model, the influencing factors of rural financial efficiency in Hebei Province are analyzed from five aspects: rural economic environment, farmers' living standards, urbanization level, rural credit level, and financial service support. The innovation lies in that by collecting relevant data, the DEA method is mainly used to calculate the superefficiency value of rural financial efficiency in Hebei Province, and the influencing factors of rural financial efficiency in Hebei Province are analyzed. The rural financial efficiency of Hebei Province has been deeply analyzed. Based on this, policies and measures to improve the rural financial efficiency of Hebei Province are proposed, which can provide a reference for the continued promotion of rural finance and the formulation and implementation of reform policies of financial institutions.

## 2. Theories and Methods of Financial Efficiency Evaluation

### 2.1. Theoretical Basis

#### 2.1.1. Theory of Rural Financial Market

In the 1980s, McKinnon and Shaw put forward the theory of the rural financial market based on financial inhibition and financial deepening. This theory holds that the rural financial system and rural economic development play a mutually promoting role. In other words, the rural financial system will restrict the development of the rural economy; on the contrary, the optimization and improvement of the rural financial system depend on the development of the rural economy. Therefore, to promote the benign development between rural finance and the rural economy, it is urgent to deepen the rural financial reform and avoid the adverse impact of the administration on the rural financial market. The rapid development of internet technology in recent years has laid a good foundation for the application of rural financial services. However, the application of internet-based financial services in rural areas has encountered difficulties due to insufficient supply and a poor cognitive environment. Liang and Chen [8] proposed countermeasures to optimize the development of network finance, promote agricultural production, improve farmers' lives, and promote rural development. Microfinance is critical for the development and poverty alleviation of microenterprises. However, microenterprises also face various obstacles while accessing microfinance services, and microfinance is not widely accepted due to misunderstandings among many stakeholders. Jalil [9] explored the impact of microfinance on the sustainable development of rural microenterprises in Malaysia. Furthermore, digital finance was integrated into a conceptual model to further study its mediating effects. Data were collected from 563 rural microenterprises using a structured questionnaire, followed by statistical analysis. The findings show that microfinance has a positive and substantial impact on the development of rural microenterprises. Moreover, digital finance mediates this relationship to a certain extent.

The article "Application of Three-Stage DEA Model Combined with BP Neural Network in Microfinancial Efficiency Evaluation" was published in 2022. Journal: Comput Intell Neurosci.

The above analysis of the rural financial market theory shows that new rural financial institutions are necessary and reasonable and provides a solid theoretical basis for the study of new rural financial institutions. The development of new rural financial institutions has stimulated the enthusiasm of small and microenterprises and farmers to participate in financial projects, such as investment, loan, and savings, and made up for the lack of financial services, insufficient financial supply, and few outlets of financial institutions in rural areas. Therefore, the new rural financial institutions promote the healthy and stable development of the rural financial market and reform China's rural financial market [10–12].

#### 2.1.2. Theory of Imperfectly Competitive Markets in Rural Finance

Stieglitz originally proposed the theory of imperfectly competitive markets in rural areas. This theory believes that the competition in the rural financial market is not sufficient and is an imperfectly competitive market. As a lender, rural financial institutions do not fully understand the borrower's situation. The lack of information will lead to the failure of the rural financial market. Proper use of some measures can avoid the disappointment in the rural financial market, such as the borrower's organization and the local government's administrative intervention [13]. Problems such as adverse selection and moral hazards caused by insufficient rural financial market information can also be effectively solved. The government encourages some farmers' financial organizations, such as mutual funds and borrowers' joint insurance groups [14]. Through the administrative assistance of the government, farmers and financial institutions in the rural financial market have achieved information equivalence, improved the operational efficiency of the rural financial market, and made the market competition in the rural financial market more complete and complete.

The article "Application of Three-Stage DEA Model Combined with BP Neural Network in Microfinancial Efficiency Evaluation" was published in 2022. Journal: Comput Intell Neurosci.

The theory of imperfectly competitive markets in rural finance proves the necessity of new rural financial institutions. The rural financial market has been in a state of incomplete competition for a long time. Therefore, most farmers in rural areas prefer long-established financial institutions such as Rural Credit Cooperatives, Postal Savings Banks of China, and Agricultural Bank of China. The new rural institutions have changed the competition pattern of the rural financial market, enriched the investment categories and composition structure of the rural financial system, expanded the financial market coverage, and improved the financial service level in rural areas [15, 16].

#### 2.1.3. DEA Model

The DEA is an efficiency analysis method proposed by American operations researcher Charnes in 1978. Using this method, the relative efficiency of a multiinput and multioutput system can be effectively measured. After the improvement and supplementation by scholars, a whole set of method systems has been gradually developed, which has been widely used in the measurement of efficiency. The DEA method is based on relative efficiency. Its principle is to determine the relatively effective production frontier under the premise of ensuring that the input and output of a set of homogeneous decision-making unit (DMU) remain unchanged. Each DMU is projected onto the production frontier, and the relative effectiveness of the DMU is evaluated by comparing the distance between the DMU and the production frontier.

The DEA method is a nonparametric analysis method, which has obvious advantages in scientific research. First, when using this method to evaluate relative efficiency, there is no need to determine the functional relationship between input and output in advance, to avoid errors that may be caused by artificially setting the functional form. Second, the DEA model automatically assigns the optimal weight to each indicator according to the actual data of input and output, without setting any weight assumptions, and has strong objectivity. Third, since the dimensions of the input and output indicators do not affect the optimal efficiency index of the DMU, there is no need for dimensionless processing. Based on the actual needs of scientific and technological financial efficiency measurement, the DEA model has unparalleled advantages.

The article "Application of Three-Stage DEA Model Combined with BP Neural Network in Microfinancial Efficiency Evaluation" was published in 2022. Journal: Comput Intell Neurosci.

#### 2.1.4. Superefficiency DEA Theory

The DEA method is a linear programming method first proposed in 1978. It has been widely used in the evaluation of production unit efficiency. The DEA evaluates the method that compares the performance of the selected indicators to assess the efficiency. Therefore, the index efficiency calculated by the DEA method is the relative efficiency, that is, the ratio of output to the input of decision-making units (DMUs). The DEA model uses the linear programming method to establish a nonparametric envelope frontier. The DMUs on the production frontier are called the effective DEA units, and the efficiency value of this unit is 100%. The DMUs not on the boundary are called invalid DEA units, and the efficiency is less than 100% [17–20].

We assume that the number of DMUs is *n*, and each decision-making unit DMU_*j*_*j*=1,2,…, *n* includes *m* inputs and *n* outputs. Let the input and output of DMU_*j*_ be *X*_*j*_ and *Y*_*j*_, respectively, where *X*_*j*_=(*x*_1*j*_, *x*_2*j*_,…,*x*_*wj*_)^*T*^, and *Y*_*j*_=(*y*_1*j*_, *y*_2*j*_,…*y*_*sj*_)^*T*^. The input-output efficiency of *DM*  *U*_*j*_ can be expressed as equation (1).

(1) $$\begin{array}{c} K_{j}=\frac{u^{T}Y_{j}}{v^{T}X_{j}},j=1,2,\ldots ,n. \end{array}$$

In equation (1), *v*^*T*^ represents the weight of input; *u*^*T*^ refers to the weight of output. Since the efficiency value cannot be greater than 1, the mathematical programming of equations (2) and (3) is established.

(2) $$\begin{array}{c} Maxu^{T}\frac{Y_{j}}{v^{T}X_{j}}, \end{array}$$

(3) $$\begin{array}{c} S.t.\frac{u^{T}Y_{j}}{v^{T}X_{j}}\leq 1,u\geq 0,v\geq 0,j=1,2,\ldots ,n. \end{array}$$

Equations (2) and (3) are converted into linear programming to obtain obtained the A. Charnes & W. W. Cooper & E. Rhodes (CCR) model, as shown in equations (4)–(6).

(4) $$\begin{array}{c} \text{Min}\theta_{0}, \end{array}$$

(5) $$\begin{array}{c} S.t.\sum_{j=1}^{n}\lambda_{j}X_{j}-\theta_{o}X_{j0}\leq 0, \end{array}$$

(6) $$\begin{array}{c} \sum_{j=1}^{n}\lambda_{j}Y_{j}\geq Y_{jo}\lambda_{j}\geq 0,j=1,2,\ldots ,n. \end{array}$$

Among equations (4)–(6), *θ*_0_ denotes the input-output efficiency value of *DM*  *U*_*j*0_; *X*_*j*0_ and *Y*_*jo*_ represent the input and output vectors of *DM*  *U*_*j*0_, respectively; and *λ*_*j*_ stands for the weight value of *DM*  *U*_*j*0_. If *θ*_0_ < 1, *DM*  *U*_*j*0_ is an invalid DEA unit; if *θ*_0_=1, *DM*  *U*_*j*0_ is a valid DEA unit.

The article "Application of Three-Stage DEA Model Combined with BP Neural Network in Microfinancial Efficiency Evaluation" was published in 2022. Journal: Comput Intell Neurosci.

Equations (7)–(10) describe the Banker & Charnes & Cooper (BCC) model suitable for variable conditions of returns to scale.

(7) $$\begin{array}{c} \text{Min}\theta_{0}, \end{array}$$

(8) $$\begin{array}{c} S.t.\sum_{j=1}^{n}\lambda_{j}X_{j}-\theta_{o}X_{j0}\leq 0, \end{array}$$

(9) $$\begin{array}{c} \sum_{j=1}^{n}\lambda_{j}Y_{j}\geq Y_{jo}, \end{array}$$

(10) $$\begin{array}{c} \sum_{j=1}^{n}\lambda_{j}=1,\lambda_{j}\geq 0,j=1,2,\ldots ,n. \end{array}$$

According to the above equations, the BCC model adds the constraint assumption ∑_*j*=1_^*n*^*λ*_*j*_=1 to the CCR model. The CCR model and the BCC model are only suitable for the comparison of DMUs with an efficiency value of less than 1 but cannot compare DMUs with an efficiency value of 1.

A superefficiency DEA model is formed by extending the DEA model. This model sorts all effective DEA units after excluding their influence when calculating the DMUs at the efficiency frontier. In other words, the evaluated DMUs are not included in the reference set when considering them. The input of the DMUs with an efficiency value of 1 increases according to a certain proportion to keep its efficiency at a specific value. This proportion is the superefficiency value. The superefficiency DEA model based on the CCR model is defined as equations (11)–(13).

(11) $$\begin{array}{c} \text{Min}\theta_{0}, \end{array}$$

(12) $$\begin{array}{c} S.t.\sum_{j=1,j\neq 0}^{n}\lambda_{j}X_{j}-\theta_{o}X_{jo}\leq 0, \end{array}$$

(13) $$\begin{array}{c} \sum_{j=1,j\neq o}^{n}\lambda_{j}Y_{j}\geq Y_{jo},\lambda_{j}\geq 0,j=1,2,\ldots ,n. \end{array}$$

When the superefficiency value of the DMU is not less than 1, the DEA is effective. For effective DMUs, if the proportion of increased input is less than the superefficiency value, its own effectiveness will not change [21, 22].

### 2.2. Backpropagation Neural Network (BPNN) Model

#### 2.2.1. Overview of BPNN

The BPNN is an artificial intelligence (AI) technology operated on a computer. It is a complex nonlinear network. The principle is to simulate the physiological process of human brain reflex. It is composed of a large number of interconnected “neurons.” It is an AI technology that can mine potential logic from a large amount of data and can autonomously explore the nonlinear relationship between data. It is a multilayer BPNN through the backpropagation of errors algorithm. Rumelharth and McCelland proposed the concept of BPNN at the end of the 20th century, which can autonomously mine internal connections through the process of data input and output, and does not need to set operation-related functions in advance. The use of the deviation gradient descent method enables the BPNN to automatically adjust the threshold of the network and the proportion of each level through the repeated correction of the deviation, and the deviation is controlled within the previously set accuracy range.

The article "Application of Three-Stage DEA Model Combined with BP Neural Network in Microfinancial Efficiency Evaluation" was published in 2022. Journal: Comput Intell Neurosci.

The training process of BPNN using a large amount of data is divided into the following stages: the first stage is the “data input” process, from the input layer to the training and learning of the hidden layer, and then to the simulation output of the output layer. Next, from the output layer through the hidden layer to the input layer, the gap between the expected output and the actual output is narrowed, and the weights and thresholds of the “reverse error transfer” stage are gradually corrected; the second stage is the iterative learning process; and the third stage is the robust training process for the desired accuracy. The application fields of BPNN are very wide, including the prediction of the price trend of financial derivatives, the warning of corporate credit risk, the prediction of the efficiency of industrial chain management, etc. By intelligently learning the inherent logic between data, many problems that require high labor costs can be efficiently solved.

#### 2.2.2. Principle of the BPNN

The BPNN consists of the input layer, output layer, and hidden layer. This model is realized based on the BP algorithm. The data are input into the network structure, and the result is output after the processing of three layers. In the forward propagation process of the BPNN, it is necessary to ensure that the nodes of each layer are independent of each other, and different levels can only affect the nodes of the forward or backward section. When the expected error and output result exceed the acceptable range, the backpropagation mechanism of the BPNN will be excited, and the error signal will return according to the propagation direction. After continuously determining the neuron connection value, the expected and output result errors will reach the ideal effect [23, 24].  Figure 1 displays the specific network structure.

#### 2.2.3. Algorithm Process of the BPNN

The BP algorithm process includes the forward propagation data process, BP error signal process, and adjustment process of internal coefficients in the hidden layer. The forward propagation data process principally consists of three steps [25]. First, the hidden layer node's data input is determined, as shown in equation (14).

(14) $$\begin{array}{c} R_{j}=\sum_{i=1}^{n}w_{ij}-\theta_{j},\left(j=1,2,\ldots ,p\right). \end{array}$$

In equation (14), *R*_*j*_ represents the input data; *θ*_*j*_ stands for the range value of neurons in the hidden layer; *w*_*ij*_ refers to the interaction coefficient between the neuron *i* in the input layer and the neuron *p* in the hidden layer; and *j* represents the number of neuron nodes in the hidden layer.

The article "Application of Three-Stage DEA Model Combined with BP Neural Network in Microfinancial Efficiency Evaluation" was published in 2022. Journal: Comput Intell Neurosci.

Then, the data output from the hidden layer nodes are calculated according to equation (15).

(15) $$\begin{array}{c} Z_{j}=f\left(R_{j}\right)=\frac{1}{1+e^{-R_{j}}},\left(j=1,2,\ldots ,p\right). \end{array}$$

In equation (15), *Z*_*j*_ signifies the output data.

Finally, the calculation method of the hidden layer calculates the output data of the output layer node.

The following describes the BP error signal process [26]. Equation (16) indicates the variance between the ideal output and the actual output to evaluate the error value of the output result.

(16) $$\begin{array}{c} e_{i}=\frac{1}{2}\sum {\left(d_{i}-Z_{i}\right)}^{2}. \end{array}$$

In equation (16), *d*_*i*_ represents the ideal value of the output result, and *Z*_*i*_ denotes the actual output of the network model.

This paragraph introduces the adjustment process of the inner coefficients in the hidden layer. The internal coefficients of nodes in different layers are adjusted in the BP process of the error signal to observe whether the error between the ideal output result and the actual output is within an acceptable range. The trained BPNN model is valid if the error is within this range, ending the training process. If the error is not within the set accuracy, then the inner coefficients in the hidden layers need to be modified again [27, 28]. First, the input increment in the hidden layer is set by equations (17) and (18).

(17) $$\begin{array}{c} \Delta w_{jt}=-\alpha \frac{\partial e_{t}}{\partial w_{jt}}\\ =-\alpha \frac{\partial e}{\partial R_{t}}\frac{\partial R_{t}}{\partial w_{jt}}=-\alpha \left(Z_{t}-d_{t}\right)Z_{t}\left(1-Z_{t}\right)y_{t}, \end{array}$$

(18) $$\begin{array}{c} \Delta \theta_{t}=-\alpha \frac{\partial e_{t}}{\partial \theta }\\ =-\alpha \frac{\partial e_{t}}{\partial R_{t}}\frac{\partial R_{t}}{\partial \theta }=-\alpha \left(Z_{l}-d_{t}\right)y_{t}\left(1-Z_{t}\right) \end{array}$$

In equations (17) and (18), *α* is a constant; Δ*w*_*jt*_ refers to the corrected weight value; and Δ*θ*_*t*_ represent the corrected threshold value.

The article "Application of Three-Stage DEA Model Combined with BP Neural Network in Microfinancial Efficiency Evaluation" was published in 2022. Journal: Comput Intell Neurosci.

Then, the increment is added to the hidden layer according to equations (19) and (20).

(19) $$\begin{array}{c} \Delta w_{\ddot{\sigma }}=-\beta \frac{\partial e_{i}}{\partial w_{\ddot{\sigma }}}\\ =-\beta \frac{\partial e_{i}}{\partial R_{j}}\frac{\partial R_{j}}{\partial w_{\ddot{\sigma }}}\\ =-\beta \frac{\partial e_{i}}{\partial Z_{j}}\frac{\partial Z_{j}}{\partial R_{j}}\frac{\partial R_{j}}{\partial w_{ij}}\\ =-\beta \frac{\partial e_{i}}{\partial Z_{j}}\left(1-Z_{i}\right)x_{i}, \end{array}$$

(20) $$\begin{array}{c} \delta_{j}=-\frac{\partial e_{i}}{\partial R_{j}}\\ =-\frac{\partial e_{i}}{\partial Z_{j}}Z_{i}\left(1-Z_{i}\right)\\ =y_{i}\left(1-Z_{i}\right)\sum \delta_{i}w_{ji}. \end{array}$$

Then, there are equations (21)–(24).

(21) $$\begin{array}{c} \Delta w_{i}=\beta \delta_{i}x_{i}, \end{array}$$

(22) $$\begin{array}{c} \Delta \theta_{j}=\beta \delta_{j}, \end{array}$$

(23) $$\begin{array}{c} w_{ij}^{\prime }=w_{ij}+\Delta w_{ij}, \end{array}$$

(24) $$\begin{array}{c} \theta_{j}^{\prime }=\theta_{j}+\Delta \theta_{j}. \end{array}$$

In the above equations, *β* refers to constant. The parameter values of the network model are iteratively calculated under the new process coefficients. This calculation is repeated until the final error value satisfies the set accuracy range, and the training process is ended at this time.

The comprehensive evaluation process through the BPNN primarily includes the following four steps. Step 1: we set the initialization parameters of the model, such as threshold, initial weight, and maximum training times. Step 2: we collect the input value of the model by normalizing the data values of each evaluation index. Step 3: we adjust the neuron parameters according to the error between the actual and expected output results. Then, we continue the iterative calculation until the obtained parameter results meet the preset conditions and the training process is ended [29–31].  Figure 2 reveals the specific algorithm flow.

The topology of the BPNN is presented in Figure 3.

The topology of BPNN includes the input layer, hidden layer, and output layer. The BPNN, that is, the learning process of the backpropagation of errors algorithm, is composed of two processes: forward propagation of information and backpropagation of errors. Each neuron in the input layer is responsible for receiving input information from the outside world and passing it to each neuron in the middle layer. The middle layer is the internal information-processing layer, which is responsible for information transformation. According to the requirements of information change capability, the middle layer can be designed as a single hidden layer or a multihidden layer structure. The information transmitted to the neurons of the output layer by the last hidden layer is further processed. After processing, the processing process of a learning forward propagation is completed, and the information processing result is output to the outside world from the output layer. When the actual output does not match the expected output, it enters the backpropagation stage of the error. The error passes through the output layer, corrects the weights of each layer according to the method of error gradient descent, and transfers back to the hidden layer and the input layer layer-by-layer. The cycle of forward propagation of information and backpropagation of errors is the process of continuously adjusting the weights of each layer, and it is also the process of BPNN learning and training. This process has been carried out until the error of the network output is reduced to an acceptable level or the up to the set number of learning times.

The article "Application of Three-Stage DEA Model Combined with BP Neural Network in Microfinancial Efficiency Evaluation" was published in 2022. Journal: Comput Intell Neurosci.

## 3. Static Efficiency Evaluation of Rural Finance Based on DEA

The efficiency of rural finance in China is studied here via the DEA method by referring to the relevant reference documents on the setting of efficiency input-output indicators of financial institutions in China. This study sets three evaluation indicators after comprehensively considering the current situation of rural finance in Hebei Province: input index, output index, and DMU [32, 33].

The DMUs are six cities in Hebei Province, namely, Hengshui, Langfang, Chengde, Zhangjiakou, Xingtai, and Shijiazhuang. To a certain extent, rural financial efficiency can reflect the contribution of rural finance to the economy. This study selects financial indicators as input indicators and economic indicators as output indicators after referring to the index selection principles in the relevant literature and comprehensively considering the availability of financial data in Hebei Province.

The input indexes include the number of fixed assets invested in the financial industry in the rural areas of each city, the number of agricultural loans in each town, the number of employees in the rural financial sector in each city, and the financial support for agriculture in each city. Among them, the financial support for agriculture represents the government economic indicators provided by local governments. The number of employees in the rural financial industry reflects the human resource status of the financial sector, which determines the level of economic development in various regions to a certain extent.

Output indexes include per capita consumption of rural households, per capita net income of rural households, and per capita gross domestic product of each city. The three indicators reflect the living and income standards of rural residents in each region and the economic development status of each area.  Figure 4 illustrates the specific index settings.

The article "Application of Three-Stage DEA Model Combined with BP Neural Network in Microfinancial Efficiency Evaluation" was published in 2022. Journal: Comput Intell Neurosci.

## 4. Evaluation of Rural Poverty Alleviation Efficiency Based on the BPNN

### 4.1. Sample Selection

This section selects S County in Hebei Province as the research object. The number of impoverished villages in this county ranks 4th among counties and districts in Hebei Province, and the number of poor populations ranks 11th. The BPNN model reported here contains 19 input values and only one output vector, and the evaluation value of mode operation efficiency. A random questionnaire survey is carried out in the poverty-stricken areas in S County, and 200 valid questionnaires are finally recovered. The 160 samples are used as the training sample set of the neural network, and the remaining 40 samples are used as the test data for network simulation.  Figure 5 displays the evaluation index system.

In Figure 5, starting from social goals, economic goals, and ability goals, the model is comprehensively considered according to the theory of multidimensional poverty and rural financial market theory so that the index setting can achieve the functions of detection, description, evaluation, and prediction. An evaluation index system is established based on the four subjects of the government, financial institutions, industry, and farmers. The first is social goals. First, the government, as the leader of each participant, controls the direction of financial support for industrial poverty alleviation. The government's realization of poverty alleviation goals is closely related to the establishment of risk sharing, compensation mechanisms, and benefit linking mechanisms for poverty alleviation projects. Second, the realization of poverty alleviation goals means reducing the occurrence of poverty, improving the living standards of farmers, and improving production conditions and infrastructure construction. The second is the economic goal; the bank is the “storage center” of the funds of this poverty alleviation model and is the main channel for farmers to obtain loans. The survey of farmers' satisfaction with the “bank's participation in the poverty alleviation and development model of the financial support industry” is mainly conducted from the aspects of the working ability, service attitude, and credit product satisfaction test of bank service personnel. Profitability is an important prerequisite for the sustainable development of financial institutions, while the repayment willingness of farmers and the bank's follow-up inspection are the basic guarantees for the bank to recover the loan and maintain profitability. The third is the ability goal. The first is the ability of industrial development, which is a vital basis for completing the task of poverty alleviation and is very important to achieve poverty alleviation and prosperity. Including product sales channels, industrial scale, industrial structure, and brand strength all determine the level of industrial development. The sustainable development of the rural economy is inseparable from the development of local industries. The second is the development ability of farmers, the improvement of income levels, and the provision of jobs, and whether to acquire new skills is crucial for farmers.

The article "Application of Three-Stage DEA Model Combined with BP Neural Network in Microfinancial Efficiency Evaluation" was published in 2022. Journal: Comput Intell Neurosci.

### 4.2. Questionnaire Design

Farmers are the judges and ultimate beneficiaries of financial support for industrial poverty alleviation. Therefore, after establishing the index system, it is necessary to investigate the understanding and satisfaction of farmers on various indicators. A five-point Likert scale is used to evaluate the satisfaction of farmers. Values from 1 to 5 represent “very poor,” “relatively poor,” “average,” “relatively good,” and “very good.” The higher the score, the higher the satisfaction degree.

### 4.3. Normalization Processing

After analyzing the index system, it can be found that it is impossible to uniformly measure each index. Therefore, the sample data need to be normalized before it is input into the neural network model to unify the measurement standard. The sample data are mapped to [0, 1], conducive to improving the performance and convergence speed of the model. The data are normalized as shown in equation (25).

(25) $$\begin{array}{c} \bar{x_{i}}=\frac{x_{i}-\bar{x_{\min}}}{x_{\max}-x_{\min}}\times d_{1}+d_{2}. \end{array}$$

In equation (25), *x*_max_ and *x*_min_ refer to the maximum and minimum values of the input sample data; $\bar{x_{i}}$ stands for the normalized sample data; and *d*_1_ and *d*_2_ equal 0.998 and 0.001, respectively.

## 5. Empirical Analysis

### 5.1. Evaluation Results of Rural Financial Efficiency Based on DEA

#### 5.1.1. Comprehensive Efficiency Analysis Based on the CCR Model

The DEAP 2.1 software is used to measure the comprehensive efficiency of rural finance in Hengshui, Langfang, Chengde, Zhangjiakou, Xingtai, and Shijiazhuang in Hebei Province from 2011 to 2020.  Figure 6 provides the results.

According to Figure 6, before 2015, the comprehensive efficiency of Xingtai, Hengshui, Shijiazhuang, and Langfang shows a downward trend. It is almost stable at around 0.95, indicating that rural finance in Hebei Province has developed steadily in recent years. The overall efficiency of rural finance has been improved to some extent. Therefore, Hebei Province's financial reform has achieved specific results. The annual average comprehensive efficiency of Hengshui, Langfang, Chengde, Zhangjiakou, Xingtai, and Shijiazhuang in Hebei Province from 2011 to 2020 is shown in Figure 7.

The article "Application of Three-Stage DEA Model Combined with BP Neural Network in Microfinancial Efficiency Evaluation" was published in 2022. Journal: Comput Intell Neurosci.

In Figure 7, among the six cities, the annual average comprehensive efficiency of Chengde is 1, indicating that it is at the frontier of efficiency and has achieved the effective DEA units. Comparing the average yearly value of comprehensive efficiency of various cities with the average value, it is found that the comprehensive efficiency of Chengde, Langfang, Zhangjiakou, and Shijiazhuang is higher than the average value. Xingtai has the lowest comprehensive efficiency value, which is only 0.649, followed by Hengshui with a value of 0.747. It shows that 74.7% of the resource input in Hengshui has achieved output, while the remaining 25.3% has not been reasonably utilized, resulting in a waste of resources. On the whole, the financial efficiency value of Hebei Province has been improved to a certain extent, but the development of various cities is not balanced.

The annual average values of comprehensive efficiency of various cities suggest significant differences in developing different cities in Hebei Province. The gap between Chengde, which has an efficiency value of 1, and Xingtai, which has the lowest efficiency value, is noticeable, leading to the low efficiency of rural finance in Hebei Province. Because of the imbalance of regional development, the cities with low efficiency represented by Xingtai and Hengshui should improve their resource utilization efficiency, minimize the gap between cities, and promote the economic development of Hebei Province by enhancing the resource rate.

#### 5.1.2. Efficiency Evaluation Based on the Superefficiency DEA Model

Although the DEA method can determine whether the efficiency value of the DMU is 1, it also has limitations. In particular, it cannot compare the efficiency values of the DMUs that have reached DEA efficiency and cannot judge which city has a higher efficiency value in the best efficiency. To solve this problem, this study introduces the superefficiency DEA model to compare the DMUs with an efficiency value of 1.  Figure 8 provides the detailed results.

The superefficiency DEA model recalculates the cities with a DEA-calculated efficiency value of 1 according to a certain proportion.  Figure 8 suggests apparent differences in the superefficiency values of cities that have reached DEA effectiveness after measurement by the DEA model. The calculation results of the DEA model show that the efficiency value of Hengshui, Langfang, and Chengde in Hebei Province in 2020 is 1, all reaching the DEA effectiveness. However, the superefficiency values of Hengshui, Langfang, and Chengde in Hebei Province in 2020 are not the same, which are 1.335, 1.336, and 1.327, respectively. In addition, there are significant differences in the superefficiency values of various cities in Hebei Province, which has caused an imbalance in rural development in Hebei Province.

The article "Application of Three-Stage DEA Model Combined with BP Neural Network in Microfinancial Efficiency Evaluation" was published in 2022. Journal: Comput Intell Neurosci.

### 5.2. Evaluation of Operational Efficiency of the BPNN Model

Each evaluation index value of the operation efficiency of the financial support industry poverty alleviation development model is used as the input vector of the neural network model, and the operation efficiency evaluation result of the model is used as the output vector. The larger the output result, the better the operation efficiency of the model. The training process ends when the training error reaches the set range by continuously adjusting the neural network's weights.

The key to explaining the evaluation results of mode operation efficiency lies in setting evaluation criteria. The research develops the evaluation standards by citing the evaluation standards set by Wu Qingtian and divides the corresponding evaluation intervals based on the equal interval length grades, as shown in Table 1 [34].

After the function and related parameters of the neural network are set, the BPNN toolbox in the MATLAB software is used to train 160 sample data. After training many times, when the sum of squares of network error meets the error target of 0.001, the training process of the BPNN is completed.

After the model training is completed, the remaining 40 sample data are substituted for the simulation verification of the model. The specific operations are as follows. The sample data are normalized and input into the trained BPNN model. The results show that the error between the expected and output values is less than 0.05. The specific results are shown in Figure 9.

After completing the training process of the BPNN, the average values of 100 randomly selected questionnaire indicators are input into the network for simulation training.  Figure 10 provides the average value of each indicator of the operation efficiency of the financial support industry poverty alleviation development model.

According to the average value of each index of the questionnaire, the operation efficiency evaluation result of the financial support industry poverty alleviation development model is 0.6995, in the interval (0.6, 0.8). In addition, the model operation efficiency is brilliant, indicating that the financial support industry poverty alleviation development model has achieved good results and promoted the development of poor rural areas.  Figure 11 reveals the local industrial development in recent years.

The article "Application of Three-Stage DEA Model Combined with BP Neural Network in Microfinancial Efficiency Evaluation" was published in 2022. Journal: Comput Intell Neurosci.

According to Figure 11, the industrial scale of S County has gradually expanded in recent years. The industrial output value has increased from 2.5 billion CNY in 2015 to 12 billion CNY in 2020, and the total industrial base is also expanding. This phenomenon shows that the financial support industry poverty alleviation development model has promoted the poverty alleviation and rural revitalization of S County and has played a specific role in promoting the development of poor rural areas in S County.

Alberca and Parte [35] took 44 internet financial listed companies as the research objects, and based on the data disclosed by the listed companies from 2015 to 2018, they explored the performance evaluation system of internet financial companies through index screening and scoring models. A total of 14 financial indicators and nonfinancial indicators were determined, and a performance evaluation indicator system for listed internet financial companies was constructed. The data of 44 listed Internet financial companies are selected, normalized, and tested for correlation, and the weights of indicators at all levels are obtained by using the analytic hierarchy process (AHP), and the expected output of the BPNN is obtained. Finally, the constructed BPNN performance evaluation model is used for network training and simulation analysis. Among them, 152 data of 38 companies in the past 4 years are selected as training samples, and the data of 6 companies in the past 4 years are used as test samples to analyze the results of simulation output. The evaluation results manifest that the comprehensive performance level of Oriental Fortune is the highest, and the comprehensive performance level of Zhongke Jincai is the lowest. The comprehensive performance level of several internet finance companies has formed obvious echelon differences. The comprehensive performance evaluation value of the five internet finance companies has decreased year by year since 2015. It is worth mentioning that despite the stricter supervision of the internet finance industry and the overall decline in performance for several consecutive years, the second, third, fourth, and fifth in 2017 still achieved a certain growth, which indicates that the internet finance industry still has a certain room for development. Oriental Fortune's comprehensive performance score is far ahead of other companies, and it is worthy of in-depth analysis to provide ideas for the sustainable development of internet finance companies. The model can evaluate the comprehensive performance level of internet finance companies within a reasonable margin of error. However, because the understanding of technical indicators is not deep enough, it is difficult to obtain relevant data on technical indicators. Therefore, although the financial performance and nonfinancial performance of the company are considered when establishing the indicator system, the selection of nonfinancial indicators is not comprehensive enough that only considers the stability and innovation ability of the companies.

The article "Application of Three-Stage DEA Model Combined with BP Neural Network in Microfinancial Efficiency Evaluation" was published in 2022. Journal: Comput Intell Neurosci.

## 6. Conclusions

Econometrics and statistics are taken as the basis of theoretical methods to determine the evaluation indexes of rural financial efficiency and evaluate the rural economic level of Hebei Province by the DEA method. In addition, the BPNN analyzes the operation efficiency of the industry's poverty alleviation and development model. The research results demonstrate that before 2015, the comprehensive efficiency of Xingtai, Hengshui, Shijiazhuang, and Langfang shows a downward trend. After 2015, the comprehensive efficiency changes of various cities in Hebei Province tended to be stable, basically stable at around 0.95, indicating that rural finance in Hebei Province has steadily developed in recent years. The overall efficiency of rural finance has been improved to some extent. It means that Hebei Province's financial reform has achieved specific results. Establishing an index system and evaluating the status quo of rural finance efficiency in Hebei Province are of great significance for accurately understanding the development of rural finance in Hebei Province. The rural financial efficiency of Hebei Province has been deeply analyzed, and based on this, policies and measures are proposed to improve the rural financial efficiency of Hebei Province. It can provide a reference for the continued promotion of rural finance and the formulation and implementation of reform policies for financial institutions. Due to the limitation of objective conditions, this study still has limitations. Certain stages and periodicities existed in the continuous deep development and improvement of poverty alleviation. Only with sufficient investigation data and in-depth field investigation can the research conclusions be scientific. Therefore, it is necessary to continue tracking and following up the development of this model to make research more scientific and reliable.

## Figures and Tables

**Figure 1:** Structure of the BPNN.

**Figure 2:** Algorithm flow.

**Figure 3:** The topology of the BPNN.

**Figure 4:** Rural financial input and output indicators by city.

**Figure 5:** Evaluation index system of operational efficiency of the financial support industry poverty alleviation development model.

The article "Application of Three-Stage DEA Model Combined with BP Neural Network in Microfinancial Efficiency Evaluation" was published in 2022. Journal: Comput Intell Neurosci.

**Figure 6:** Overall efficiency. (a) Comprehensive efficiency of cities in Hebei Province; (b) annual average value of complete efficiency.

**Figure 7:** The annual mean value of comprehensive efficiency of various cities.

**Figure 8:** Superefficiency values of various regions.

**Figure 9:** Comparison results of expected values and output values.

**Figure 10:** The average value of each indicator.

**Figure 11:** Industrial development status of S County.

**Table 1:** Model operation efficiency evaluation criteria.

Index level	Very poor	Relatively poor	Average	Relatively good	Very good
Comprehensive evaluation value	[0, 0.2)	[0.2, 0.4)	[0.4, 0.6)	[0.6, 0.8)	[0.8, 1]

## Data Availability

The data used to support the findings of this study are included within the article.
